The article "KDELR3 Is a Prognostic Biomarker Related to the Immune Infiltration and Chemoresistance of Anticancer Drugs in Uveal Melanoma" was published in 2022. Journal: Dis Markers.

# KDELR3 Is a Prognostic Biomarker Related to the Immune Infiltration and Chemoresistance of Anticancer Drugs in Uveal Melanoma

**DOI:** 10.1155/2022/1930185

**Published:** 2022-08-21

**Authors:** Jingnan Zhang, Juan Zhang, Jing Guan, Lisha Yu, Shilong Yan

**Affiliations:** ^1^Department of Pharmacy, Linyi Central Hospital, Linyi, Shandong, China; ^2^Department of Traditional Chinese Medicine, Qingdao Eighth People's Hospital, Qingdao, Shandong, China; ^3^Department of Cataract, Jinan Aier Eye Hospital, Jinan, Shandong, China

## Abstract

Uveal melanoma (UM) is an intraocular malignancy in adults in which approximately 50% of patients develop metastatic diseases and have a poor clinical outcome. Immunotherapies are quickly becoming a need, and recent research has produced some amazing achievements in this area. In the current investigation, an attempt was made to evaluate the prognostic usefulness of KDELR3 in UM, particularly its connection with tumor-infiltrating lymphocytes (TILs). The expression patterns of mRNAs and related clinical data of 80 UM patients were obtained from The Cancer Genome Atlas (TCGA). By using RT-PCR, we were able to investigate whether or not UM cells and D78 cells expressed KDELR3. The Kaplan-Meier approach, as well as univariate and multivariate tests, was utilized in order to investigate the potential predictive significance of KDELR3 expression. The associations between KDELR3 and TILs and immunological checkpoints were analyzed in order to evaluate the effect that KDELR3 may have on UM immunotherapy. On the basis of the differential expression of KDELR3, a distribution of the half-maximal inhibitory concentration (IC50) of various targeted medicines was observed. In this study, we found that the expression of KDELR3 was distinctly increased in most types of tumors. In addition, KDELR3 was highly expressed in UM cells. Moreover, patients with high KDELR3 expression exhibited a shorter overall survival and disease-free survival than those with low KDELR3 expression. Multivariate analyses confirmed that KDELR3 expression was an independent prognostic factor for overall survival and disease-free survival in patients with UM. Furthermore, KDELR3 expression was demonstrated to be positively correlated with macrophage M1, T cell CD8, T cell follicular helper, dendritic cell resting, and T cell CD4 memory activated. Meanwhile, the expression of KDELR3 was related to several immune checkpoints. The IC50 of AP-24534, BHG712, bleomycin, camptothecin, cisplatin, cytarabine, GSK1070916, and tipifarnib was higher in the KDELR3 high-expression group. In conclusion, KDELR3 may be applied as a potential diagnostic and prognostic biomarker for UM patients.

## 1. Introduction

Uveal melanoma (UM) is the most prevalent form of intraocular cancer found in adults around the world [1]. It is a malignant tumor that begins in the melanocytes of the eye's choroid plexus, iris, and ciliary body [2]. The development of early metastases is the primary contributor to the disease' alarmingly high mortality rate [3, 4]. Because the biology behind the beginnings and spread of UM is unknown, there is currently no effective treatment available for patients who have already developed metastatic illness [5, 6]. It is estimated that almost half of UM patients will have further deterioration, and the clinical outcome for the patients remains poor [7]. The use of chemotherapy and targeted therapies typically does not result in the maintenance of long-term tumor control. Thus, immunotherapy is increasingly emerging as a potentially useful treatment option [8, 9]. Meanwhile, it is essential to investigate potential new prognostic biomarkers or therapeutic targets that are effective.

The KDEL (Lys-Asp-Glu-Leu) receptor family, also known as the KDELR family, is an important protein family that plays a role in recycling the chaperones and maintaining the dynamic balance of trafficking between the Golgi and the endoplasmic reticulum (ER) [10, 11]. Recent researches have shown evidence to imply that KDELRs are essential components of the Golgi transport control mechanism. KDELR is responsible for initiating transport via the Golgi complex after it binds to the heterotrimeric signaling G protein G (q/11), where it then activates the proteins [12, 13]. The third confirmed member of the KDEL family is referred to as KDELR3. KDELR3 expression in arteriosclerosis macrophages might be noticeably different from that in nonarteriosclerosis tissues, and the higher expression level in nonarteriosclerosis tissues, which can be used as a potential predictive factor [14]. In addition, a number of investigations have found that the expression of KDELR3 was markedly aberrant in a variety of malignancies, including hepatocellular carcinoma and prostate adenocarcinoma [15, 16]. However, its expression and clinical significance in UM have not been investigated.

The vast majority of immune system components have been linked to both the beginning and the development of UM [17]. In the context of tumor immunity, tumor cells serve the function of antigens, and immune cells and leukocytes penetrate the tumor tissue via chemotaxis in order to mount an immunological defense [18, 19]. In addition, immune evasion is a significant contributor to the development of tumors. At the moment, a wide variety of novel immunotherapies are being utilized in UM, some of which are PD-1, PD-L1, and CTLA-4 inhibitors [20–22]. However, these methods are only useful for a small number of individuals, and the vast majority of patients have either a limited or nonexistent response to the treatment, particularly when the UM is in a more advanced stage. Therefore, in order to investigate the potential diagnostic application of new biomarkers, it is necessary to perform exhaustive studies on the association that exists between key genes and overall survival in UM.

In the present investigation, we began by conducting pan-cancer assays, and we discovered that the level of KDELR3 was noticeably elevated in the majority of different kinds of cancers. After that, we discovered that the level of KDELR3 expression was considerably elevated in UM cells. In addition, we investigated the expression of KDELR3 in UM and investigated the connection between the level of KDELR3 expression and the prognosis of patients with UM. Finally, exhaustive bioinformatics studies were carried out in order to investigate the underlying mechanisms of KDELR3. This study contributes to the following individualized diagnosis and treatment of UM by providing relevant information.

## 2. Materials and Methods

### 2.1. Cell Lines and Culture

The uveal melanoma cell lines (MUM-2C, OCM-1A, MUM-2B, and C918) and one melanocyte cell line (D78) were purchased from purchase Chinese Academy of Sciences (Beijing, China). DMEM was used as the medium for the cultivation of D78, OCM-1A, and MUM-2C, while RPMI 1640 was utilized for the upkeep of C918 and MUM-2B.

### 2.2. RNA Isolation and RT-PCR

Extraction of total RNAs from grown cells was carried out using TRIzol (Life Technologies) in accordance with the procedure provided by the manufacturer. cDNAs were reverse transcribed using HiScript III Reverse Transcriptase (Vazyme) using oligo (dT) and random hexamers, then qRT-PCR analysis was performed on them, and then they were put through PCR and qPCR analysis. Real-time quantitative PCR was carried out using ChamQ SYBR qPCR Master Mix (Vazyme) and either a 7900HT Fast Real-Time PCR System or an ABI Prism 7900HT Real-Time PCR System (Applied Biosystems). The relative expression of genes was quantified to GAPDH. The primer sequences were presented as follows: KDELR3 5′-TCCCAGTCATTGGCCTTTCC-3′ (forward) and 5′-CCAGTTAGCCAGGTAGAGTGC-3′ (reverse) and GAPDH 5′-GGAGCGAGATCCCTCCAAAAT-3′ and 5′-GGCTGTTGTCATACTTCTCATGG-3′.

### 2.3. Data Resource and Preprocessing

The GDC Data Transfer Tool was used to retrieve the RNA expression profiles of 80 UM patients from TCGA database in FPKM format. In addition, mRNA and lncRNA expression data were also retrieved. On the UCSC Xena website, the pertinent clinicopathological characteristics, such as sex, age, and cancer stage, were retrieved.  Table 1 contains an in-depth presentation of the clinical features.

### 2.4. Functional Enrichment Analysis

We separated the samples from TCGA datasets into two groups based on the median expression level of KDELR3 and screened the dysregulated genes between the two groups using the “limma” program [23]. This was done so that we could gain a deeper understanding of the underlying mechanism of KDELR3. Then, we examined the genes in the two groups using the Gene Ontology (GO) and the Kyoto Encyclopedia of Genes and Genomes (KEGG) assays to see if they were abundant in significant biological processes. Then, we used the “http://org.Hs.eg.db” package to convert the gene symbols into Entrez IDs, and we used the “cluster Profiler,” “ggplot2,” and “enrich plot” packages to conduct a pathway enrichment analysis for the DEGs based on the GO database and KEGG. This was done by combining the results of the pathway enrichment analysis with the DEGs. After applying the false discovery rate (FDR) approach, the *P* values were recalculated, and significantly enriched pathways were determined to have an FDR of 0.25 or lower.

### 2.5. Tumor-Infiltrating Immune Cells (TICs) Profile

Using the LM22 signature, the CIBERSORT algorithm was utilized to conduct an analysis of the percentage of immune cells that had penetrated the tumor microenvironment (TME) [24]. The LM22 signature, which consists of 547 genes, was utilized to detect 22 different types of immune cells that had infiltrated the tissue. In addition, we investigated the difference between KDELR3 expression and the immune cells that had penetrated the TME by performing difference and correlation analysis.

### 2.6. Correlation Analysis

The Cancer Regulome Explorer (http://explorer.cancerregulome.org/) enables users to search, filter, and visualize analytical results generated from TCGA data and explore associations among heterogeneous features. On the chromosomal level, we utilized it to display the expression of KDELR3 as well as its association with other variables that are associated with malignancies. In order to investigate the degree of association that exists between KDELR3 and immunological checkpoints, a Pearson's analysis was carried out. The “pheatmap” tool in R was used to present the results of the analysis.

### 2.7. IC50 Score

When determining the efficacy of a medicine or the response of a sample to treatment, one of the most essential indicators to look at is the half-maximal inhibitory concentration, also known as the IC50. The sample-based transcriptome, which makes use of the Genomics of Drug Sensitivity in Cancer (GDSC) database, which is the biggest publicly available pharmacogenomics resource, can predict the response of each sample to the targeting and/or immunotherapy of UM.

### 2.8. Statistical Analysis

Statistical analysis was performed in R v. 4.0.2 (R Core Team, Massachusetts, USA) and GraphPad Prism v. 8.01 (GraphPad Software, La Jolla, CA, USA). The Wilcoxon rank-sum test was utilized in order to carry out analyses on box plots. Spearman's coefficient was utilized in order to carry out the correlation study. In order to investigate the nature of the connection that exists between KDELR3 expression levels and clinicopathological characteristics, both the chi-square and *t*-tests were carried out. The Kaplan-Meier method was utilized in the construction of the survival curves (log-rank test). Survival data were evaluated through the univariate and multivariate Cox regression analysis. A *p* < 0.05 was deemed to be statistically significant.

## 3. Results

### 3.1. The mRNA Expression of KDELR3 in Cancers

In order to determine whether or not KDELR3 expression was correlated with cancer, we analyzed its levels in a variety of tumors as well as the normal tissues. Data from TCGA datasets showed that KDELR3 mRNA expression was distinctly higher in ACC, BLCA, BRCA, CESC, CHOL, COAD, DLBC, ESCA, GBM, HNSC, KIRP, LIHC, LUAD, LUSC, OV, PAAD, PRAD, PEAD, SARC, SKCM, STAD, THCA, THYM, UCEC, and UCS tumor specimens compared to that in normal specimens, suggesting that it could serve as a tumor promoter in the progression of diverse tumors (Figure 1(a)). Nevertheless, TCGA datasets did not contain any normal uveal specimens. Therefore, it is unknown whether KDELR3 demonstrated a dysregulated behavior in UM. Therefore, we utilized RT-PCR to investigate the level of KDELR3 in D78 cells and four different UM cell lines. We discovered that the level of KDELR3 expression was noticeably elevated in UM cells in comparison to D78 cells (Figure 1(b)).

### 3.2. Correlation of KDELR3 Expression with Clinicopathological Features

Further investigation into the relationship between KDELR3 and the clinicopathological features of UM was carried out so that we could determine the clinical significance of KDELR3 in UM. The patients diagnosed with UM were separated into two groups based on the mean expression of KDELR3 (high KDELR3 expression group and low KDELR3 expression group). As exhibited in Table 1, our investigation revealed that the level of KDELR3 was not connected to any clinical parameters, including age, gender, or stage (*p* > 0.05).

### 3.3. The Prognostic Value of KDELR3 Expression in UM

After that, we used the Kaplan-Meier method to determine whether or not the levels of KDELR3 expression can accurately predict the prognosis of patients with UM. Patients who had high levels of KDELR3 expression had a shorter overall survival (Figure 2(a), *p* < 0.001) and disease-free survival (Figure 2(b), *p* < 0.001) than those who had low levels of KDELR3 expression. These findings were demonstrated by statistical analysis. Time-dependent ROC analysis indicated the prognostic accuracies were 0.798 at 1 year, 0.888 at 3 years, and 0.887 at 5 years, respectively (Figure 2(c)). In order to assess whether the KDELR3 expression level was an independent factor for prognostic prediction in UM patients, both univariate and multivariate analyses were carried out. We observed that KDELR3 expression was an independent prognostic factor for overall survival (HR = 13.397; 95% CI: 3.931-45.657; *p* < 0.001, Table 2) and disease-free survival (HR = 17.116; 95% CI: 3.961-73.971; *p* < 0.001, Table 3) in patients with UM.

### 3.4. Function Enrichment Analysis of DEGs

Our group evaluated dysregulated genes in UM specimens that were in the high KDELR3 expression group in order to gain a better understanding of the role that KDELR3 plays in UM. Then, we utilized these genes in GO and KEGG analyses that we carried out.  Figure 3(a) contains a list of the top 30 most enriching GO terms. In BP, the DEGs were mainly associated with RNA catabolic process, mRNA catabolic process, establishment of protein localization to membrane, translational initiation, and viral gene expression. In CC, they were related to mitochondrial inner membrane, cell-substrate junction, focal adhesion, ribosome, and ribosomal subunit. In MF, the DEGs mainly involved in cadherin binding, ubiquitin-like protein ligase binding, ubiquitin protein ligase binding, structural constituent of ribosome, and ribonucleoprotein complex binding. The results of KEGG assays revealed that the most distinctly enriched biological processes included pathways of neurodegeneration-multiple diseases, amyotrophic lateral sclerosis, Alzheimer's disease, Parkinson's disease, Huntington's disease, prion disease, and thermogenesis (Figure 3(b)).

### 3.5. Correlation Analysis between KDELR3 Expression and Infiltrating Immune Cells

TIICs are a crucial component of the intricate microenvironment that plays a role in regulating the development and progression of numerous malignancies [25, 26]. Survival rates from cancer can be accurately predicted based on factors such as the number of lymphocytes that infiltrate the tumor and their activity level. As a result, we investigated whether or not there was a connection between immune cell infiltration and KDELR3 expression. We explored the relationship of KDELR3 expression and immune infiltration level based on CIBERSORT in order to identify whether KDELR3 expression was connected with the immune infiltration level in a variety of malignancies. The results indicated that KDELR3 expression was positively associated with macrophage M1, T cell CD8, T cell follicular helper, dendritic cell resting, and T cell CD4 memory activated, while negatively associated with NK cell resting, B cell naïve, eosinophils, neutrophils, monocytes, mast cell resting, and T cell CD4 memory resting (Figure 4). According to the results of our research, the level of immune infiltration in UM was directly proportional to the amount of KDELR3 expression.

### 3.6. Correlation Analysis between KDELR3 Expression and Immune Checkpoint Molecules in UM

Subsequently, we determined the linear correlation between the expression of immune checkpoint related genes (CD86, PDCD1, CD48, CD80, CD276, TNFSF18, TNFRSF8, and TNFRSF18) and risk scores using Spearman's rank correlation coefficient. These genes include CD86, PDCD1, CD48, CD80, CD276, TNFSF18, TNFRSF8, and TNFRSF18. The results indicated that the expression of immunosuppression-related genes had positive correlation with KDELR3 expression in TCGA datasets (Figure 5).

### 3.7. IC50 Score

When determining how well patients may respond to targeted medication therapy, IC50 is an essential metric to use [27, 28]. We were able to predict changes in the IC50 scores of chemotherapeutic drugs between different KDELR3 expression groups by using data from GDSC. The IC50 of AP-24534, BHG712, bleomycin, camptothecin, cisplatin, cytarabine, GSK1070916, and tipifarnib was higher in the KDELR3 high-expression group (Figure 6). Therefore, these data demonstrate that there was a statistically significant difference in the distribution of IC50 values for targeted drugs among the different KDELR3 expression groups.

## 4. Discussion

UM is a malignant primary intraocular tumor that affects adults at a higher rate than any other type of malignant primary intraocular tumor [29]. The majority of UM are often treated with surgery or radiotherapy, which typically results in survival rates that are comparable over the short term [30, 31]. Because of its unique biology and clinical behavior, around fifty percent of patients will be given a bad prognosis, which may include disease recurrence and dissemination. To date, conventional methods have not been able to provide a survival benefit or exact prognostic prediction for these patients. On the other hand, more recent systemic treatments, in particular immunotherapies and targeted therapy, have dramatically improved patient survival. Nevertheless, the discovery of novel prognostic indicators was of utmost significance for patients diagnosed with UM. In this work, we conducted a retrospective analysis to choose biomarkers that linked with the immunological milieu of the tumor in order to predict prognosis and identify the segment of the population that would benefit the most from immune checkpoints.

The role of KDELR3, which was only recently shown to be associated with tumors, was seldom ever mentioned. The KDELR3 gene is a member of the KDEL endoplasmic reticulum protein retention receptor family. Its product, KDELR3, is translated into proteins. According to the findings of the study carried out by Marie and colleagues, the inhibition of KDELR3 led to a reduction in the amount of melanoma cells that colonized the lungs during experimental metastasis assays. This was accomplished by modulating the activity of the metastasis suppressor KAI1 [32]. However, the expression and clinical significance of KDELR3 in UM have not been investigated. In this study, the mRNA expression of KDELR3 was shown to be significantly greater in the majority of different tumors, which suggested that it may play a role as an oncogenic molecule in the development of a variety of different malignancies. When compared with D78 cells, the level of KDELR3 in UM cells was found to be noticeably higher thanks to the findings of RT-PCR. In patients diagnosed with UM, we found that the level of KDELR3 expression acted as an independent predictive factor for both overall survival and survival free of illness. In general, the results of our study revealed that KDELR3 could be a predictive biomarker for UM patients.

We carried out a GO and KEGG function enrichment analysis using the genes that were dysregulated between the high KDELR3 expression group and the low KDELR3 expression group in order to gain a deeper understanding of the possible role that KDELR3 played in the progression of tumors. Our findings suggested that KDELR3 may play an important role in the progression of neurodegeneration-multiple diseases, amyotrophic lateral sclerosis, Alzheimer's disease, Parkinson's disease, Huntington's disease, prion disease, and thermogenesis.

Cancer tissues consist of not only malignant neoplastic cells but also immune cells, fibroblasts, endothelial cells, and an abundant collection of cytokines, chemokines, and growth factors [33]. The TME is formed by these components and their complex interaction with one another. The various cellular compartments that make up the TME are able to critically regulate tumorigenesis, which is essential not only to tumor initiation, malignant progression, and metastasis but also to response to therapy [34, 35]. In the TME, the majority of host cells that are drawn to and activated are immune cells. Determining appropriate immunotherapy treatment plans for cancer patients now relies significantly on the detection of immune cells that can serve as biomarkers in the cancer immunological microenvironment. The quantity of immune cells and how they are distributed is the single most critical element in determining the eventual course of a tumor, including whether or not it will inhibit or promote carcinogenesis, cell metastasis, cell migration, and tumor angiogenesis [36, 37]. Nevertheless, the immunological microenvironment in the many forms of cancer is intricate and heterogeneous. In this study, we found that KDELR3 expression was positively associated with macrophage M1, T cell CD8, T cell follicular helper, dendritic cell resting, and T cell CD4 memory activated, while negatively associated with NK cell resting, B cell naïve, eosinophils, neutrophils, monocytes, mast cell resting, and T cell CD4 memory resting. According to the findings that we obtained, the level of immune infiltration in UM was directly proportional to the amount of KDELR3 expression. In recent years, immune checkpoint blockade therapy has emerged as one of the most important immunotherapies for the treatment of cancers. This therapy is credited for fundamentally altering the landscape of cancer treatment. Inducing a long-lasting anticancer response and removing a block in the immune system are the goal of immunotherapy that blocks immunological checkpoints [38, 39]. In addition, we discovered that the expression of genes linked to immunosuppression had a positive connection with the expression of KDELR3 in TCGA datasets. When determining how well patients may respond to targeted medication therapy, IC50 is an essential metric to use. We were able to predict changes in the IC50 scores of chemotherapeutic drugs between different KDELR3 expression groups by using data from GDSC. The IC50 of AP-24534, BHG712, bleomycin, camptothecin, cisplatin, cytarabine, GSK1070916, and tipifarnib was higher in the KDELR3 high-expression group. Consequently, these findings showed that the IC50 distributions of targeted drugs in distinct KDELR3 expression groups were statistically significant.

However, despite the fact that we conducted an exhaustive and methodical study on KDELR3, we found nothing. This study has certain caveats and restrictions to it. First, the findings were based on data that was collected in the past, and more data collected in the present was required to prove the clinical relevance of it. Second, experiments in vivo and in vitro are required to validate our findings about the possible functions of KDELR3. If these experiments are successful, the credibility of our findings will be significantly increased. Third, despite the fact that KDELR3 expression was highly connected to immune cell infiltration and the prognosis of human malignancies, we do not have any direct proof that KDELR3 played a role in immune infiltration and hence influenced the prognosis. Therefore, the methods via which KDELR3 participated in immune modulation are still a mystery, and the precise pathway needed additional research.

## 5. Conclusions

Our research contributed to a better understanding of the potential function of KDELR3 mRNA in tumor immunology as well as its relevance as a prognostic indicator. It was found that the levels of KDELR3 mRNA connected with both the prognosis and the immune infiltration levels in UM, indicating that it can be employed as a biomarker for predicting the outcome of the disease. It is necessary to investigate the possibility that KDELR3 inhibitors would cause interference with immune cells.

## Figures and Tables

**Figure 1:** KDELR3 expression levels in human cancers. (a) Using data from TCGA database, GEPIA was able to assess the levels of KDELR3 expression in a variety of tumor types. (b) RT-PCR was utilized in order to investigate whether KDELR3 was expressed in MUM-2C, OCM-1A, MUM-2B, C918, and D78.

**Figure 2:** Prognostic value of KDELR3 expression in UM patients. (a, b) In TCGA datasets, Kaplan-Meier survival curves and log-rank tests were performed on high-risk and low-risk score groups. (c) The AUC for 1-, 2-, and 3-year overall survival in TCGA datasets.

**Figure 3:** Enrichment analysis in TCGA UM cohort. (a) Gene ontology enrichment. (b) Kyoto Encyclopedia of Genes and Genomes pathway analyses.

**Figure 4:** Analysis of the correlation between the amount of KDELR3 expression and the amount of immune infiltration.

**Figure 5:** The differential expression of immune checkpoint molecules in TCGA cohorts between the high-risk group and the low-risk group.

**Figure 6:** Distribution of IC50 scores of targeted drugs in different KDELR3 expression groups via ACLBI website.

**Table 1:** Correlation between tissue KDELR3 expression level and clinicopathological characteristics.

Characteristic	Low expression of KDELR3	High expression of KDELR3	*p*
*n*	40	40	
Pathologic T stage, *n* (%)			0.644
T2	8 (10%)	6 (7.5%)	
T3	17 (21.2%)	15 (18.8%)	
T4	15 (18.8%)	19 (23.8%)	
Pathologic N stage, *n* (%)			0.579
N0	28 (35.4%)	24 (30.4%)	
NX	12 (15.2%)	15 (19%)	
Pathologic M stage, *n* (%)			0.128
M0	28 (35.9%)	23 (29.5%)	
M1	0 (0%)	4 (5.1%)	
MX	12 (15.4%)	11 (14.1%)	
Pathologic stage, *n* (%)			0.113
Stage II	22 (27.8%)	17 (21.5%)	
Stage III	18 (22.8%)	18 (22.8%)	
Stage IV	0 (0%)	4 (5.1%)	
Gender, *n* (%)			1.000
Female	17 (21.2%)	18 (22.5%)	
Male	23 (28.7%)	22 (27.5%)	
Age, *n* (%)			0.502
≤60	22 (27.5%)	18 (22.5%)	
>60	18 (22.5%)	22 (27.5%)	
Age, mean ± SD	57.95 ± 14.03	65.35 ± 13	0.017

**Table 2:** Univariate and multivariate analysis of the associations of overall survival with various clinicopathologic parameters and KDELR3 expression in uveal melanoma patients.

Characteristics	Total (*N*)	Univariate analysis		Multivariate analysis	
		Hazard ratio (95% CI)	*p* value	Hazard ratio (95% CI)	*p* value
Pathologic T stage	80				
T2	14	Reference			
T3	32	3.138 (0.401-24.558)	0.276		
T4	34	4.572 (0.590-35.428)	0.146		
Pathologic N stage	79				
N0	52	Reference			
NX	27	0.890 (0.360-2.198)	0.800		
Pathologic M stage	78				
M0	51	Reference			
M1 and MX	27	0.924 (0.373-2.287)	0.865		
Pathologic stage	79				
Stage II	39	Reference			
Stage III and stage IV	40	1.502 (0.629-3.585)	0.360		
Age	80				
≤60	40	Reference			
>60	40	2.123 (0.914-4.933)	0.080	2.528 (1.055-6.061)	**0.038**
Gender	80				
Female	35	Reference			
Male	45	1.542 (0.651-3.652)	0.325		
KDELR3	80				
Low	40	Reference			
High	40	12.517 (3.685-42.512)	**<0.001**	13.397 (3.931-45.657)	**<0.001**

**Table 3:** Univariate and multivariate analyses of the associations of progression-free survival with various clinicopathologic parameters and KDELR3 expression in uveal melanoma patients.

Characteristics	Total (*N*)	Univariate analysis		Multivariate analysis	
		Hazard ratio (95% CI)	*p* value	Hazard ratio (95% CI)	*p* value
Pathologic T stage	80				
T2	14	Reference			
T3	32	2.512 (0.314-20.124)	0.386		
T4	34	4.433 (0.572-34.338)	0.154		
Pathologic N stage	79				
N0	52	Reference			
NX	27	0.985 (0.391-2.483)	0.974		
Pathologic M stage	78				
M0	51	Reference			
M1 and MX	27	1.024 (0.405-2.585)	0.961		
Pathologic stage	79				
Stage II	39	Reference			
Stage III and stage IV	40	1.607 (0.640-4.033)	0.312		
Age	80				
≤60	40	Reference			
>60	40	1.872 (0.785-4.461)	0.157		
Gender	80				
Female	35	Reference			
Male	45	1.351 (0.558-3.275)	0.505		
KDELR3	80				
Low	40	Reference			
High	40	17.116 (3.961-73.971)	**<0.001**	17.116 (3.961-73.971)	**<0.001**

## Data Availability

The data used to support the findings of this study are included within the article. Further inquiries can be directed to the corresponding author.
